# Ghanaians Might Be at Risk of Inadequate Dietary Intake of Potassium

**DOI:** 10.1155/2016/3150498

**Published:** 2016-12-06

**Authors:** David Oscar Yawson, Michael Osei Adu, Benjamin Ason, Frederick Ato Armah, Emmanuel Boateng, Reggie Quansah

**Affiliations:** ^1^Department of Soil Science, School of Agriculture, College of Agriculture and Natural Sciences, University of Cape Coast, Cape Coast, Ghana; ^2^Department of Crop Science, School of Agriculture, College of Agriculture and Natural Sciences, University of Cape Coast, Cape Coast, Ghana; ^3^Soil Research Institute, Council for Scientific and Industrial Research, Accra, Ghana; ^4^Department of Environmental Science, School of Biological Science, College of Agriculture and Natural Sciences, University of Cape Coast, Cape Coast, Ghana; ^5^Department of Biological, Environmental & Occupational Health Sciences, School of Public Health, College of Health Sciences, University of Ghana, Accra, Ghana

## Abstract

Adequate dietary intake of potassium (K) helps fight noncommunicable diseases (NCDs), mainly hypertension and cardiovascular diseases. This paper (i) estimated the K intake of Ghanaian population using food supply and food composition data and (ii) compared this estimate with the WHO recommended requirement for K in order to assess if there is a risk of inadequate K intake. Food supply data (1961–2011) was obtained from the FAO Food Balance Sheet (FBS) to derive trends in food and K supply. The average food supply in the FBS for 2010 and 2011 was used in assessing the risk of inadequate dietary intake of K. The K contents of the food items were obtained from food composition databases. The mean K supply per capita per day was approximately 856 mg. The assessment suggests a potentially large risk of inadequate dietary K supply at both individual and population levels. The results suggest the need for assessing options for managing K deficiency, including assessment of K supplying power of soils and K fertilizer management in food crop production systems, as well as empirical estimates of K content of food items (including those underreported in the FBS) and mixed diets in Ghana.

## 1. Introduction

Potassium (K) is an essential element which plays crucial roles in the nutrition and health of plants, animals, and humans. Potassium is known to activate over 60 enzymes in plants, promotes photosynthesis, plays a role in stomata opening, use of nitrogen, transport of assimilates, and microbial population in the rhizosphere [1–3]. Major roles of K in humans and animals include maintenance of water balance, osmotic pressure and acid-base balance, activation of enzymes, mediation of carbohydrate, and protein metabolism. More importantly, potassium plays a crucial role in the regulation of neuromuscular activity and heartbeat [4, 5].

Inadequate intake of vitamins and mineral elements (known as the “hidden hunger”) has adverse health outcomes and is a global health and food security challenge. As a result, hidden hunger has received increased policy, research, and practical attention, especially with regard to vitamin A, iron, iodine, zinc, and selenium [6]. Globally, noncommunicable diseases (NCDs) constitute a major contributor to mortality and morbidity [7, 8]. There is a strong evidence of association between low K intake and increased risk of a number of NCDs, including hypertension, cardiovascular disease, chronic kidney stone formation, and low bone-mineral density [4, 9–12]. Hypertension is a major risk factor for cardiovascular diseases, notably coronary heart disease and stroke [9]. Yet, the instrumental role of adequate K intake, through food, and its cost-effectiveness in combating the global burden of NCDs is only beginning to attract priority attention [9].

In Ghana, hypertension is a major public health problem [13]. Between 1988 and 2007, the number of new cases of hypertension reported in public health facilities increased from 49,087 to 505,180 [14]. Crude prevalence of hypertension in Ghana (based on 140/90 mmHg threshold) is between 25% and 48%, with higher prevalence in urban populations [13]. Hypertension is the second leading cause of outpatient morbidity (after malaria) in the Greater Accra Region [14]. Stroke and hypertension are among the leading causes of hospital admission and death in Ghana [13]. Hypertension has been identified as an important cause of heart and renal failure in Ghana [15, 16].

Due to its moderating role in hypertension and cardiovascular diseases, K-rich diets (especially fruits and vegetables) are now highly recommended to reduce high blood pressure [17]. However, the reported average K intake from diets in several countries is below recommended levels [9]. Diets are the main source of K intake in humans. The K content of food components largely derives from the soils on which feed and food crops are grown. Yet, the K status of soils and fertilizer management in most agroecosystems continue to receive less attention, and this is particularly so in Ghana [3, 5]. To draw attention to the need to pay much attention to K flows from farm to fork, this paper therefore assessed the risk of insufficient dietary supply of K in adult Ghanaian population using food supply and composition data.

## 2. Methods

### 2.1. K Supply from Foods

Prevalence of K deficiency can be assessed directly via the analysis of urine or blood samples. In the absence of such analysis and for larger population size, the deficiency of K can be quantified via food surveys or dietary analysis using food composition data [18] even though food surveys data can be biased by systematic misreporting and behavioural change [19]. Where there is paucity of data on representative food surveys or food composition tables, as is the case for Ghana, alternative sources of data such as the Food Balance Sheet (FBS) provided by the Food and Agriculture Organization (FAO) can be used to indirectly quantify the adequacy of K intake as has been done in similar studies (e.g., [20, 21]). Hence, the current study used the FBS data to indirectly quantify the risk of inadequate K intake in Ghana. A FBS provides a snapshot of the supply and uses of about 92 food items/groups for each of FAO member countries during a given reference period [22]. The FBS has supply and utilization sides. For a given reference period and food item, total supply is the sum of total domestic production and imports, adjusted to changes in stocks that might have occurred since the beginning of the reference period. On the utilization side, the total supply of the given food item is decomposed into quantities exported, used for animal feed and seed, processed for food and nonfood uses, losses, and the fraction available for human consumption [22, 23]. The fraction of supply of the food item available for human consumption is divided by the total population of a given country to obtain the* per capita supply*. Thus, the FBS does not directly provide information on food consumption but on food availability, which was used as a proxy for consumption in the current study.

The average food supply per person for the latest years (2010 and 2011) in the FBS was computed. This was done to capture minimum interannual variation in food availability or consumption. Food items were selected from the FBS based on the kg food supply per person. The dietary K supply per person was estimated as the product of per capita food supply (based on the FBS) and the K content of the food items [24, 25]. The K content or supply of each food component was calculated using the corresponding conversion factors for the edible fraction provided in the food composition table. The K contents of the food components (except for cocoa and products, oats, crustaceans, cephalopods, and other molluscs) were obtained from the West African Food Composition Table [26]. The K contents of the food items that were not found in West African Food Composition Table [26], such as cocoa and products, were obtained from the United States Department of Agriculture-Agricultural Research Service (USDA-ARS) Nutrient Database for Standard Reference [27]. This method has been applied previously in studies that estimated the adequacy or otherwise of minerals in the diets of populations in some countries (see [6, 21, 24, 25, 28]).

To build the final database of K contents of selected food items, food items were excluded if the product of supply and K content was zero or if that particular food component is not known to be widely or commonly consumed in Ghana according to local knowledge. In the food composition databases, effort was made to identify the categories of food items that best matched those in the FBS [25]. Where two or more categories of the same food items are consumed in Ghana according to local knowledge, an average K content was computed to represent that food item (see Table 2). The total K supply (or intake) per person was calculated as the sum of the products of food supply and K composition of all the food items as described earlier. All K contents or concentration data are expressed as mg 100 g^−1^ fresh weight edible portion. The per capita food supply and associated K supply for the period 1961–2011 were computed using the FBS and the food composition table, with a similar approach as described earlier, to obtain the trends.

### 2.2. Adequacy of K Supply from Food

The likely risk of inadequate dietary supply of K was assessed at the individual level, and then the prevalence of deficiency at population level was estimated using the EAR cut-point approach [24, 25, 29]. A detailed description of this approach, its strengths, and assumptions are provided in Food and Nutrition Board [29]. Due to paucity of information, the recommended K intake for adults, 3510 mg K per person per day [9], was used in the current study as the reference nutrient intake (RNI). The RNI represents the intake level of a mineral which meets the nutrient requirements of 97.5% apparently healthy individuals in a population group for a given age and sex [25]. Again, due to paucity of information, we used a standard conversion of RNI 1.2*∗*EAR (as Joy et al. [25] used for Mg and explained by Allen et al. [30]) to convert the RNI to an estimated average requirement (EAR) of 2925 mg.

To assess the risk of inadequacy at the individual level, the EAR value was used to represent the “required mean K intake” (*r*), while the total K supply (based on the FBS and food composition data) represented the “observed mean intake” (*y*). The difference between *y* and *r*, *D*, gives an initial impression of the adequacy or otherwise of K intake per person. To allow a probability of correct conclusion on the adequacy of intake, the magnitude and direction (positive or negative) of the ratio of *D* and its standard deviation (SD_*D*_) were estimated [29]. SD_*D*_ represents the daily variation in individual intake of K. To calculate SD_*D*_, the standard deviation of the required intake (SD_*r*_) was estimated at 10% and 15% [29], while the pooled standard deviation of the observed intake (SD_*i*_) for adult males and females was obtained from reference tables [29] due to lack of national-level data. SD_*D*_ was then calculated using the procedure in [29].

(1) $$\begin{array}{c} {SD}_{D}={\left[\;\frac{{SD}_{i}^{2}}{n}+{SD}_{r}^{2}\;\right]}^{1/2}, \end{array}$$

where *n* is the number of days of observed intake data.

Subsequently, the ratio of *D* to SD_*D*_ was computed for each case (at 10 and 15% for adult males and females) to obtain the probability of correct conclusion regarding the adequacy or otherwise of individual intake (based on interpretation table in [29]).

The EAR cut-point method was used to estimate the likely prevalence of inadequate intake at the population level. In the EAR cut-point method, a normal distribution of daily intake among the population was expected. The proportion of the population at risk of inadequate intake is assumed to be equivalent to the proportion with intake below the EAR [29]. Because we only had a point estimate of dietary K supply, and following an approach used in some previous studies (e.g., [24, 25]), daily K intake in the population was assumed to have a normal distribution, centred on mean dietary supply and with a coefficient of variation (CV) of 25% or 30%. Based on this, the prevalence of inadequate K intake was estimated using the average of 2010 and 2011 population provided in the FBS which was used to calculate the per capita food supply.

## 3. Results

### 3.1. Contribution of Food Components

There were 46 food items in the Food Balance Sheet (FBS) for Ghana (Table 1). The food item coffee and products (mainly instant powder coffee) had the greatest K content (3640 mg), followed by mixed ground spices with K content of 1040 mg. “Meat, other” (mainly game meat) had the third largest K content (923 mg) while “sugar (raw equivalent)” had the least (2 mg). The top 10 values of K supply ranged from 524 (plantain) to 3640 mg. The top three K supply food items (instant powder coffee, mixed ground spices, and game meat) were consumed in very low quantities in Ghana between 2010 and 2011 according to the FBS.

The top five food items consumed in large quantities are (in order of importance) cassava and products, yams, plantains, roots (other), and rice (milled equivalent). The K supply from these food items was 264, 278, 189, 32, and 2 mg per capita per day, respectively (Table 1). These are followed by maize and products (3 mg K per cap per day) and tomatoes and products (38 mg K per cap per day). Total K intake from food supply per person was approximately 856 mg per day. Of this, starchy roots contributed 84% while vegetables contributed only 5% (Figure 1(a)). The rest contributed approximately 2% or less. Oranges and mandarins contributed 50% of the total contribution of fruits (Figure 1(b)). Of the starchy roots, yams and cassava contributed the largest (Figure 1(c)). Wheat and products contributed the largest among the cereals (Figure 1(d)), while tomato and products contributed 82% of the total contribution from vegetables (Figure 1(e)). “Game meat, other” contributed 55% of the total contribution of meat, fishes, and seafood.

### 3.2. Trends in K Intake

Between 1974 and 1983, dietary intake of K declined sharply from around 600 mg to around 450 mg (Figure 2). Thereafter, K intake from food supply increased marginally and reached a plateau around 1989. However, from 1991, K intake from food supply increased consistently, with food supply, to around 900 mg.

### 3.3. Risk of Inadequate K Intake

The average dietary K supply per person for 2010 and 2011 was approximately 856 mg per day. The estimated variations in individual daily intake (SD_*D*_ at both 10% and 15%) were large for the different sex and age categories considered (Table 2). Similarly, the *D*/SD_*D*_ ratios (at both 10% and 15%) were large and negative. According to the interpretation tables provided by the Food and Nutrition Board [29], these large, negative ratios suggest a 98% probability that the usual dietary K intake of the individual is inadequate. This potentially large risk of K deficiency at the individual level suggests a potentially large probability of deficiency at the population level, making the assessment of population-level prevalence of deficiency needless. Notwithstanding, using the EAR cut-point method with a CV of 25% and 30% (based on average population of 24,542 million for 2010 and 2011) resulted in a risk of deficiency for the entire population.

## 4. Discussion

Based on food supply and composition data, dietary K intake at both individual and population levels in Ghana, between the years 2010 and 2011, was much lower than recommended by WHO [9]. This suggests a potential large risk of K deficiency in the Ghanaian adult population for the years under consideration. Because K is largely supplied from diets and is highly absorbable (about 85–90%), K deficiency is thought to be rare. However, K is also easily lost from the human body through excreta and sweat [4]. The risk of K deficiency is just beginning to get the requisite attention due to its role in noncommunicable diseases, which are among the leading causes of morbidity and mortality globally. The K intake in several countries has been found to be below recommended levels [9]. Not surprisingly, the results in the current study show a potentially widespread risk of deficiency in dietary intake of K in adult Ghanaian population.

Dietary source of potassium largely depends on the K status and fertilizer management of the soils on which crop plants for human and animal feed are grown. The results in this study show that yams, cassava, and plantains contributed the bulk of dietary energy and K supply. This directs attention to K management in food crop production, as well as the quality of diets. While cassava is more widely consumed in larger quantities and is a good source of K, cassava is largely grown on marginal lands by smallholder farmers, with almost zero fertilizer input. In Ghana, fertilizer application largely focuses on nitrogen and phosphorus supply. It is normally assumed that the soils have good K supplying power. However, based on a study on K dynamics in representative soils of Ghana, Yawson et al. [3] reported that K fertilizer application might be necessary even on soils thought to be rich in K. Roots and tubers are heavy K feeders and can rapidly reduce the K supply of even K-rich soils after a few years of continuous cultivation. Cassava is widely grown in the southern part of Ghana, largely in forest zones where split and frequent K fertilizer application might be necessary [3]. On the other hand, yams are grown mainly in the savanna and transitional zones where less frequent but large K fertilizer application might be required to saturate the exchangeable pool and make K immediately available to crops [3]. Hence, Ghana ought to begin to pay attention to K management in its food cropping systems. Both the total amount required (quantity) and the frequency of application need urgent attention.

With quality of diets, the deliberate consumption of fruits and vegetables is only beginning to increase due to health awareness programmes; but even this is constrained by cost, availability and traditional eating habits. The gradual increase in the consumption of fruits and vegetables might be countered by a parallel increase in the consumption of processed foods and westernized diets, especially in urban centres. Moreover, in urban settings, rice (which is lower in K than starchy roots) is increasingly becoming the dominant staple [31], a situation that might have resulted in large contribution of rice to dietary energy but low contribution to K intake in Ghana. Although Ghana is a leading producer of premium cocoa in the world, the consumption of cocoa products in Ghana is low due to cost and eating habits. There is the need for empirical studies on K contents of Ghanaian food crops (especially staples) and mixed diets and its relationship with the high incidence of hypertension observed in urban settings [13–15].

The limitations of the approach adopted in the current study have been acknowledged by previous studies (e.g., [6, 24, 25]). The accuracy of data in the FBS and the food composition databases will affect the accuracy of the current estimate. The data fed to the FAO FBS might be unreliable due to Ghana's poor data collection and aggregation on food production, import, and export. There can also be the issue of underreporting regarding the scale of consumption of some food items. For example, Ghanaians are known to consume large quantities of game meats (bush meat) and other nontimber forest products (NFTPs) which are rich in K; yet this is likely underestimated in the FBS. Similarly, Ghanaians are known to consume appreciable amounts of “molluscs, other,” mainly snails and squids, but the FBS does not report food items that are not commercially declared. In Ghana, bush meat is the second most widely eaten meat after chicken [32, 33]. Key examples of bush meat and other NFTPs commonly eaten in Ghana include grasscutter, antelope, rats, bats, snails, mushrooms, and honey [34]. In 2014, the Wildlife Division of the Forestry Commission of Ghana estimated the annual domestic trade in bush meat alone at US$ 140 million [35]. While this estimate excludes nontraded (commercially undeclared) bush meat, it suggests that consumption of bush meat can be quite high in Ghana. Similarly, coastal communities have access to a range of fish at different periods that might not be reported. Due to the underreporting of these food items not considered to be “mainstreamed” or obtained from other sources such as subsistence farming or from the wild, the estimated risk of inadequate K intake can deviate from reality. Hence, the result here must be interpreted with caution as it might not reflect the true dietary K intake or serum K in the population.

## 5. Conclusion

The risk of K deficiency is just beginning to get attention due to the role of K in the global burden of noncommunicable diseases such as hypertension and cardiovascular disease. Based on FBS data and food composition databases, the current study shows potentially large risk of inadequate dietary K intake at both individual and population levels among adult Ghanaian population. Cassava and yams contributed the bulk of dietary K supply. While the result in the current study ought to be interpreted with caution, it provides indications for policy attention. The findings suggest the need for empirical assessment of K management in food crop systems and the K content of food crops and mixed diets in Ghana. It also suggests the need for studies on K deficiency at a larger scale.

## Figures and Tables

**Figure 1:** Contribution of food items to total K supply for Ghana based on 2010-2011 average food supply data.

**Figure 2:** Trend in daily per capita K in food supply and per capita food supply in Ghana for the period 1961–2011.* Mean daily capita* ^−*1*^ *K content (primary axis, filled black circles with continuous line); food supply in Ghana (secondary axis, filled grey squares with broken line).*

**Table 1:** Estimated 2010-2011 average food supply and potassium composition of 46 edible Food Balance Sheet (FBS) items for Ghana.

Food category	Commonly eaten food/product in Ghana	K (mg)	Kg/cap/yr	K/cap/yr	K/cap/day
Wheat & products	Bread, wheat, white	117.00	17.64	2063.30	5.65
Rice (milled equivalent)	Rice, white, polished, boiled (without salt)	20.10	32.40	651.01	1.78
Maize & products	Maize, white, stiff porridge (without salt)	40.00	27.11	1084.20	2.97
Oats^*∗*^	Oats, regular and quick, unenriched, cooked with water (including boiling and microwaving), without salt	70.00	0.16	10.85	0.03
Millet & products	Millet, whole grain, boiled (without salt)	124.00	6.11	757.02	2.07
Sorghum & products	Sorghum, whole grain, boiled (without salt)	122.00	8.24	1004.67	2.75
Cassava & products	a	418.58	230.35	96417.12	264.16
Potatoes & products^*∗*^	Snack, potato chips, made from dried potatoes, plain	637.00	0.21	130.59	0.36
Sweet potatoes	Sweet potato, yellow, boiled (without salt)	369.04	5.10	1880.25	5.15
Yams	Yam tuber, boiled (without salt)	687.00	147.48	101318.76	277.59
Roots, other	b	313.43	36.99	11593.86	31.76
Sugar (raw equivalent)	Sugar	2.00	11.60	23.19	0.06
Beans/peas^*∗*^	c	300.49	0.72	215.60	0.59
Soyabeans^*∗*^	d	573.26	0.02	8.60	0.02
Groundnuts (shelled eq)	e	723.74	5.97	4317.13	11.83
Coconuts including copra	f	379.88	5.86	2224.17	6.09
Tomatoes & products	g	616.00	22.66	13955.48	38.23
Onions	h	133.95	6.23	834.49	2.29
Vegetables, other	i	241.43	8.65	2088.33	5.72
Oranges, mandarins	Orange, raw	121.18	21.46	2599.92	7.12
Lemons, limes & products^*∗*^	j	114.34	1.67	190.95	0.52
Grapefruit & products^*∗*^	k	96.18	0.03	2.89	0.01
Bananas	l	238.40	1.99	474.42	1.30
Plantains^*∗*^	m	524.20	131.24	68793.39	188.48
Apples and products^*∗*^	n	101.00	1.03	103.53	0.28
Pineapples and products	Pineapple, pulp, raw	104.65	0.99	103.61	0.28
Fruits, other	o	151.06	12.89	1946.39	5.33
Coffee & products^*∗*^	Coffee, instant, powder	3640.00	0.06	200.20	0.55
Cocoa beans & products^*∗*^	Beverages, cocoa mix, powder	712.00	3.68	2616.60	7.17
Tea (including mate)^*∗*^	Tea, infusion	18.00	0.05	0.90	0.002
Spices, other^*∗*^	Spices, mix, ground	1040.00	0.05	52.00	0.14
Beer	p	31.33	4.31	135.05	0.37
Beverages, fermented	Ovaltine beverage with skimmed milk (without sugar; fortified)	204.00	14.05	2866.20	7.85
Pigmeat	Pork, meat, approx. 40% fat, boiled (without salt)	230.77	1.04	240.00	0.66
Bovine Meat	Beef, meat, 15–20% fat, boiled^*∗*^ (without salt)	254.00	1.23	312.42	0.86
Mutton & goat meat	Goat, meat, boiled (without salt)	316.04	1.75	553.08	1.52
Poultry meat	Chicken, light meat, flesh and skin, boiled (without salt)	128.00	7.09	906.88	2.48
Meat, other	Game meat, dried	923.00	4.86	4481.17	12.28
Cream^*∗*^	q	114.50	0.02	2.29	0.01
Butter, ghee	Cheddar	82.30	0.10	7.82	0.02
Fats, animals, raw	Margarine, fortified	18.00	0.20	3.60	0.01
Eggs	r	133.64	1.17	156.36	0.43
Milk excluding butter	Milk, cow, canned, evaporated	303.00	8.67	2627.01	7.20
Fishes	s	258.05	6.28	1619.89	4.44
Crustaceans^*∗*^	t	204.00	0.08	16.32	0.04
Cephalopods^*∗*^	u	454.50	0.10	43.18	0.12
Total					**908.60**

a: cassava, tuber, boiled (without salt) & cassava, tuber, dried. b: cocoyam, tuber, boiled (without salt) & taro, tuber, boiled (without salt). c: beans, liquid from stewed kidney beans; beans, baked, home prepared; peas, edible-podded, boiled, drained, without salt; peas, edible-podded, frozen, cooked, boiled, drained, with salt; peas, green, raw & cowpea, boiled (without salt). d: soya bean, boiled (without salt) & soya bean, combined varieties, boiled (Ghana) (without salt). e: groundnut, shelled, dried, raw & groundnut paste. f: coconut, mature kernel, fresh, raw; coconut, immature kernel, fresh, raw; coconut, kernel, dried, raw & coconut water. g: tomato, red, ripe, boiled (without salt) & tomato paste, concentrated. h: onion, raw & onion, boiled (without salt). i: cocoyam, leaves, boiled^*∗*^ (without salt); amaranth leaves, boiled (without salt); cabbage, raw; carrot, raw; eggplant, boiled (without salt); garlic, raw; lettuce, raw; okra fruit, boiled (without salt); peppers, chilli, raw; pepper, sweet, red, raw; pepper, sweet, red, boiled (without salt); pepper, sweet, green, raw & pepper, sweet, green, boiled (without salt). j: lemon, raw & juice, lemon, unsweetened. k: juice, grapefruit, canned, unsweetened & grapefruit, pulp, raw. l: banana, white flesh, raw & banana, yellow flesh, raw. m: plantains, cooked; plantains, green, fried; snacks, plantain chips, salted; plantain, ripe, boiled (without salt) & plantains, ripe, fried. n: sweet apple, fruit, raw; juice, apple, canned, or bottled; apple, with skin, raw & apple, without skin, raw. o: avocado, pulp, raw; mango, deep orange flesh; mango, orange flesh, raw; papaya, fruit, ripe, raw & watermelon, fruit, raw. p: beer European (4.4% alcohol); beer, millet (est. 3% alcohol) & beer, sorghum (est. 3% alcohol). q: cream, whipping, 38% fat & cream, 13% fat. r: egg, chicken, boiled (without salt) & egg, chicken, fried. s: anchovy, fillet, steamed (without salt); mackerel, grilled (without salt and fat); mudfish, grilled (without salt and fat); sardine, steamed (without salt); tilapia, grilled (without salt and fat) & tuna, grilled (without salt and fat). t: spiny lobster, mixed species, cooked, moist heat & crab, queen, cooked, moist heat. u: octopus, common, cooked, moist heat & squid, mixed species, cooked, fried. ^*∗*^K composition was sourced from USDA National Nutrient Database for Standard Reference Software v.2.6.1. and the rest were from the FAO West African Food Composition Table. The K composition is presented as mg per 100 g edible portion.

**Table 2:** Extent of adequacy of individual K intake for different sex and age categories in Ghana based on 2010-2011 average food supply.

	Female		Male	
	19–50 years old	51+ years old	19–50 years old	51+ years old
SD_*D*10_	295.87	294.94	298.60	296.45
SD_*D*15_	441.01	440.38	442.84	441.40
*D*/SD_*D*10_	−6.82	−6.84	−6.75	−6.80
*D*/SD_*D*15_	−4.57	−4.58	−4.55	−4.57

Note: SD_*D*10_ denotes the daily variation in individual intake of K estimated at 10% standard deviation while SD_*D*15_ denotes the estimate at 15%. Values used in the calculations: required intake (2925 mg per day); standard deviations of the required intake at 10 and 15% (SD_*r*10_ and SD_*r*15_, resp.) = 292.5 mg per day and 438.75 mg per day, respectively.
